RETRACTED

# The Effect of Topical Benzydamine Hydrochloride and Cuff Pressure Monitorization on Postoperative Sore Throat Due to Intubation

**DOI:** 10.7759/cureus.53725

**Published:** 2024-02-06

**Authors:** Bilge Olgun Keleş, Menşure Kaya

**Affiliations:** 1 Department of Anesthesiology and Reanimation, Giresun University, Giresun, TUR; 2 Department of Anesthesiology and Reanimation, University of Health Science, Dr. Abdurrahman Yurtaslan Oncology Training and Research Hospital, Ankara, TUR

**Keywords:** dysphagia, hoarseness, endotracheal tube cuff pressure monitoring, benzydamine hydrochloride, postoperative sore throat

## Abstract

Objective: Postoperative sore throat (POST) is the most common discomfort after endotracheal intubation. Damage to the tracheal mucosa caused by inappropriate endotracheal tube (ETT) cuff pressure has been shown as the major factor. Monitoring the ETT cuff pressure at a certain value reduces this damage. Benzydamine hydrochloride (BH) has proven to be effective on sore throat and studies have shown that it is also effective on POST. In this study, the efficacy of BH and ETT cuff pressure monitoring on POST was evaluated.

Materials and methods: After ethics committee approval 210 patients in the ASA (American Society of Anesthesiologists) I-III risk group undergoing elective surgery were included in the study. Routine anesthesia monitoring, induction, and maintenance were provided. Patients were randomly divided into three groups. Thirty minutes before surgery, the posterior pharyngeal wall was sprayed with BH in group 1 and distilled water in groups 2 and 3. Intraoperatively, the first and second groups were monitored to keep the ETT cuff pressure between 22 and 26 cmH_2_O, while no intervention was performed in the third group. The incidence and severity of postoperative dysphagia, hoarseness, and POST were questioned.

Results: There was no difference between demographic data, and gender was not associated with POST. There was a statistically significant difference between the first and second groups and the third group in terms of all three symptoms questioned (p<0.01). No difference was observed between the first and second groups. Side effect rates were similar. Smoking was not found to be associated with symptoms.

Conclusion: The incidence and severity of POST, dysphagia, and hoarseness are reduced when the ETT cuff is inflated with a pressure of 22-26 cmH_2_O after intubation with a manometer and maintained at this pressure range throughout the operation. There was no beneficial effect of BH.

## Introduction

In general anesthesia, endotracheal intubation is a standard technique to keep the airway open, control respiration, and prevent aspiration [1]. The most common side effect is postoperative sore throat (POST). According to clinical studies, the incidence of POST varies between 14% and 75% [2]. Many factors can cause this symptom. The most crucial factor is endotracheal tube (ETT) cuff pressure. The effect of ETT cuff pressure on tracheal mucosal capillary perfusion and the duration of intubation has also been associated with POST [2,3]. It is recommended to use high-volume, low-pressure tubes during intubation and to maintain ETT cuff pressure at 22-25 cmH_2_O to minimize this side effect [4].

RETRACTED

Nitrous oxide (N_2_O), a gas anesthetic used in routine anesthesia, can quickly enter ETT cuffs and increase cuff pressure by diffusing into dead spaces [5,6]. The formation of tracheal mucosal lesions causes sore throat, hoarseness, and cough due to an increase in cuff pressure.

Benzydamine hydrochloride (BH) is a topical non-steroidal anti-inflammatory drug with additional analgesic and local anesthetic properties. Several studies have shown BH can prevent POST due to endotracheal intubation and laryngeal mask [7,8].

This study hypothesized that topical BH and ETT cuff pressure monitoring, which have been shown to be individually effective in preventing POST, would increase their effectiveness when used together.

## Materials and methods

This study was approved by the ethics committee of a tertiary teaching hospital under number 254. The patients were informed before surgery and their written informed consent was obtained. The study was conducted by the tenets of the Declaration of Helsinki. 

Study design

This is a randomized, controlled, double-blind, single-center trial of topical BHs and ETT cuff pressure monitoring at POST for intubated elective general anesthetic surgery patients. The patients were divided into three groups: group 1, group 2, and group 3.

Participants

A total of 210 adult patients aged 20-60 years with an American Society of Anesthesiologists Physical Status (ASA PS) I-III undergoing elective surgery were included in the study. Patients with a history of preoperative sore throat, non-cooperation, known allergy to BH, mallampati >3, multiple intubation attempts, head and neck surgery, and laparoscopic surgery were excluded.

Randomization

Patients were randomized by placing the computer-generated papers with the numbers one, two, and three in a sealed envelope divided into three groups. Solutions were prepared in bottles of the same color and numbered one, two, and three. BH was prepared in bottle one, distilled water was prepared in bottles two and three. The solutions were administered to the patients according to the numbers on the sealed envelopes selected by the patients. The patients and the postoperative follow-up physician were blinded to the groups.

RETRACTED

Management of anesthesia

Group 1

Four puffs (1.08 mg, 0.045 g spray 1) of BH (Tantum Verde Spray, Santa Farma, Istanbul, Turkey) were applied to the posterior pharyngeal wall 30 minutes before intubation, and ETT cuff pressure was monitored intraoperatively.

Group 2

Four puffs of distilled water were applied to the posterior pharyngeal wall 30 minutes before intubation and ETT cuff pressure was monitored intraoperatively.

Group 3

Four puffs of distilled water were sprayed on the posterior pharyngeal wall 30 minutes before intubation, but ETT cuff pressure monitoring was not performed.

Standard monitoring techniques were used in the operating theatre. Induction of anesthesia was performed with thiopental 5-7 mg/kg, fentanyl 1-2 µg/kg, and rocuronium 0.6 mg/kg. Second-year residents performed tracheal intubation. Residents were blinded to the groups. Female patients were intubated with 7 mm, and male patients with 8 mm diameter ETT (high-volume/low-pressure cuff, Tyco/Healthcare; Kendal Curity Tracheal Tube). After intubation, the ETT cuffs were connected to a pressure monitoring transducer (VBM cuff pressure measurement, VBM Medizin Technik GmbH, Germany) for group 1 and group 2. The ETT cuff pressure was inflated to 22-26 cmH_2_O and maintained at this level by assessment at 10-minute intervals. Anesthesia was maintained with 2% sevoflurane (Sevorane Abbvie S.r.l. Campoverde di Aprilia, Italia) and 70%/30% N_2_O/O_2_ with a fresh gas flow of 3 L/min.

Outcome evaluation

The primary outcome was the incidence of POST. Secondary outcomes were the severity of POST, the incidence of hoarseness, and dysphagia.

Patients' age, weight, sex, ASA, mallampati, and duration of surgery were recorded. Postoperatively, patients were assessed by a blinded physician for the presence and severity of hoarseness, dysphagia, and sore throat for 24 hours, immediately after extubation and at 1, 2, 4, and 24 hours. POST was scored on a four-point scale: 0=no sore throat, 1=mild sore throat (complaining of sore throat only when asked), 2=moderate sore throat (complaining of sore throat on its own), 3=severe sore throat (voice change or hoarseness with sore throat). Nausea/vomiting was recorded. Smokers were recorded.

Sample size

In a power analysis using G-Power 3.1.9.7 with type I error (α ) 0.05, type II error (β) 0.05, and power 80%, the sample size was calculated as 54 in each group based on data from a previous study reporting a 20% reduction in the incidence of POST between BH and saline use. Considering 20% attrition, 70 patients were included in each group [9].

RETRACTED

Statistics

Statistics were performed with IBM SPSS v23. Normality analyses of the data were performed by the Kolmogorov-Smirnov test. Quantitative data showing normal distribution were compared by independent sample t-test and ANOVA, and non-normally distributed data were compared by Mann-Whitney U and Kruskal Wallis tests. Qualitative data were compared by Pearson Chi-square test. Data were presented as mean ± standard deviation and n (%). The statistical significance value was accepted as p<0.05.

## Results

The study was completed with 210 patients (Figure 1).

**Figure 1:** CONSORT flow diagram CONSORT, Consolidated Standards of Reporting Trials; BH, benzydamine hydrochloride

The three groups had no statistically significant difference regarding demographic data, ASA, mallampati score, and duration of surgery (Table 1).

**Table 1:** Patient characteristics and duration of surgery between groups Values are presented in mean ± SD or number of patients. ASA PS, American Society of Anesthesiologists Physical Status

		Group 1 (n=70)	Group 2 (n=70)	Group 3 (n=70)	P
Age (years)		45.3 ± 11.7	46.4 ± 11.3	47.2 ± 12.4	0.644
Weight (kg)		70.9 ± 14.3	74.6 ± 13.5	70.7 ± 13.2	0.171
Female		42 (60%)	37 (53%)	40 (57%)	0.692
ASA PS	1	44 (63%)	41 (58%)	40 (57%)	0.684
	2	26 (37%)	27 (38%)	28 (40%)	
	3	0 (0%)	2 (3%)	2 (3%)	
Mallampati score	1	49 (70%)	52 (74%)	57 (81%)	0.286
	2	21 (30%)	18 (26%)	13 (19%)	
Duration of surgery (min)		139.3 ±63.4	135.8 ± 67.2	133.8 ± 57.4	0.872

POST was more severe in group 3 than in groups 1 and 2 at 0, 1, and 24 hours after extubation and this result was statistically significant between the groups (p<0.05) (Table 2). 

**Table 2:** Comparision of POST severity with groups in different time periods *difference between groups 1-3,  groups 2-3, n(%) h, hours

Time (h)	Severity	Group 1 (n=70)	Group 2 (n=70)	Group 3 (n=70)	P
0	None	88.6	82.9	45.7	<0.01*
	Mild	10.0	15.0	34.8	
	Moderate	1.4	2.1	10.1	
	Severe	0	0	9.4	
1	None	85.7	84.3	37.1	<0.01*
	Mild	10.0	10.0	35.7	
	Moderate	4.3	4.3	15.7	
	Severe	0	1.4	11.4	
24	None	88.6	82.9	34.3	<0.01*
	Mild	7.1	11.4	45.7	
	Moderate	4.3	4.3	11.4	
	Severe	0	1.4	8.6	

The incidence of POST was 14.3% in group 1, 17.1% in group 2, and 66.9% in group 3. The incidence of hoarseness was 15.1% in group 1, 17.2% in group 2, and 71.9% in group 3. The incidence of dysphagia was 15.8% in group 1, 19.0% in group 2, and 70.2% in group 3. The results were statistically significant (p<0.01) (Table 3). 

**Table 3:** Comparison of incidence of POST, hoarseness, and dysphagia between groups *difference between groups 1-3, groups 2-3, n(%) POST, postoperative sore throat

	Group 1 (n=70)	Group 2 (n=70)	Group 3 (n=70)	P
POST	14.3	17.1	66.9	<0.01*
Hoarseness	15.1	17.2	71.9	<0.01*
Dysphagia	15.8	19.0	70.2	<0.01*

There was no statistically significant relationship between smoking and symptoms. There was no significant difference between the groups in terms of the incidence of nausea and vomiting.

RETRACTED

## Discussion

In our study, ETT cuff pressure monitoring was found to effectively reduce the incidence and severity of POST. In group 3, more patients reported severe POST, hoarseness, and dysphagia compared to the other two groups. However, no significant difference was found between groups 1 and 2 and thus the effectiveness of BH on the incidence and severity of POST could not be demonstrated.

BH is a non-steroidal anti-inflammatory drug with local anesthetic, analgesic, and antibacterial properties and a terminal half-life of approximately 8 hours. BH is active in the early vascular phase of the inflammatory process. It also inhibits platelet aggregation and prostaglandin synthesis. The literature recommends BH for the treatment of acute sore throat [10-12]. Local tissue concentrations of BH have been reported to be higher with topical application than with systemic application. Absorption of BH is very rapid after systemic administration. After topical application, absorption is slower, plasma peak time is longer, and thus, its effect lasts longer [13]. The safety of BH has been demonstrated in preclinical studies, and no clinically significant side effects have been shown [7-13]. Analyzing two systematic reviews of the literature on BH and POST, BH can prevent POST and is recommended prophylactically [7,8]. There are studies in which BH was applied to the oropharynx, tracheal tube, and cuff of the tube and compared with lidocaine, dexpanthenol, ketamine, and aspirin [9,14-16]. In these trials, no site superiority was found and superior effects were observed compared with other drugs. The optimal dose, application, and timing of topical BH cannot be determined. In our study, we applied four puffs (1.08 g) to the posterior pharyngeal wall 30 minutes before intubation, which is generally recommended as the effective dose.

POST is one of the most common subjective complaints reported by patients after tracheal intubation, and the incidence in our study ranged from 14.3% to 66.9%, which is consistent with the literature. Studies show a higher incidence and severity of POST in the female gender, and others show no difference between the genders. We did not find a gender difference in sore throat in our research [2,17,18]. The causes of sore throats are multifactorial and differ between men and women. Comparing genders is not meaningful, as ETT shape and cuff pressure changes have been shown to be more important factors [19].

RETRACTED

ETT cuffs are usually checked by the traditional palpation method or inflated until no air leak is heard and then not checked until extubation. In studies where ETT cuffs were checked using a manometer, there was generally an increase in ETT cuff pressure over time [1,4,20-24]. Ünsal et al. inflated the ETT cuff of one group with 25 cmH_2_O and the other with the traditional method and then measured it without making any adjustments [24]. They showed that the pressure of the ETT cuff inflated with the palpation method was higher, and the incidence of POST was higher in this group.

The pressure of the ETT cuff is transmitted directly to the tracheal mucosa. Overinflation increases the area of contact between the cuff and the trachea. The greater the area of contact, the greater the damage to the mucosa. Damage begins when the pressure in the ETT cuff exceeds the capillary pressure in the tracheal artery. It has been shown that blood flow decreases significantly at pressures above 30 cmH_2_O and ischemic damage begins within 15 minutes at pressures above 50 cmH_2_O. If the damage persists, it can lead to severe complications such as vascular ischemia, loss of ciliary activity, inflammation, ulceration, and tracheal stenosis [1,20,21,25]. To-oru et al. and Donnely et al. in their large number of post-mortem studies in cadavers showed that mucosal ulceration was present in the tracheal specimens they examined as early as 1 hour after intubation [26,27]. Less than 10% of those intubated for less than 24 hours, but almost all of those intubated for more than 48 hours, had deep ulceration. Therefore, they emphasized that intubation time is effective, but high pressure is a more critical factor. In their meta-analysis of ETT cuff measurements, Hockey et al. found that routine cuff pressure measurement and adjustment to maintain pressure within the recommended range were the most important factors in preventing POST in the intubated patient [21]. Mami et al. monitored the ETT cuffs, which inflated to a pressure of 20 cmH_2_O in one group and 30 cmH_2_O in the other, throughout the operation and kept them the same [22]. There was no significant difference in POST between the groups. They reported that constant pressure was effective in preventing POST. In our study, we did not use a continuous pressure transducer in the groups in which we monitored the ETT cuff pressure, but we fixed the cuff pressure at 22-26 cmH_2_O at 10-minute intervals. In line with the literature, POST was lower in these groups and higher in the group where we did not monitor the cuff pressure.

N_2_O is a gas with 34 times greater solubility than nitrogen and can easily diffuse into air spaces. The ETTs we used are made of polyvinyl chloride (PVC) and have a high N_2_O permeability [5]. Koşar et al. compared N_2_O anesthesia with air anesthesia in their study [28]. They observed a rapid increase in ETT cuff pressures in the N_2_O group after the first 15 minutes and showed that the pressures increased to 45 cmH_2_O and above. The incidence of POST was higher in the N_2_O group. The same results were obtained by Jonny P et al. in laparoscopic surgery [29]. Combes et al. inflated the cuff with saline and air in N_2_O anesthesia and made a comparison [30]. While the pressures in the air group increased again, the saline-inflated group remained at constant pressure. At extubation, tracheal lesions were evaluated with an endoscope and were higher in the air group. Benesh et al. gave N_2_O anesthesia to cats in an animal experiment and showed that ETT cuff pressures increased to around 48 cmH_2_O and that tube size and flow rate did not affect the pressure increase in this study [6].

RETRACTED

In addition to cuff pressure monitoring, which was considered the most important factor when we reviewed all the studies on POST, we added BH, which is effective in many studies. In our trial, where we hypothesized that the combination of two factors in POST prevention would further reduce sore throat, we did not get the result we expected. We did not find a statistically significant difference in the incidence of POST, hoarseness, and dysphagia between group 1 with benzydamine and ETT cuff monitoring and group 2 with distilled water and ETT cuff monitoring. There was a statistically significant difference in all symptoms between group 1 with BH and cuff monitoring and group 3 with distilled water and no cuff monitoring. We interpreted the difference in favor of cuff pressure, not in favor of BH.

The limitations of our study are that we did not investigate the side effects such as dry mouth, burning, stinging, and numbness that occur immediately after application due to the use of BH.

## Conclusions

In conclusion, the main cause of POST is damage to the tracheal mucosa caused by ETT cuff pressure. Hoarseness and dysphagia also increase in parallel with sore throat. All of these symptoms can be reduced with a simple precaution.

We have shown that inflating the ETT cuff to a pressure of 22-26 cmH_2_O with a manual manometer after intubation and periodically reducing the cuff pressure to normal limits during surgery is effective in preventing POST, hoarseness, and dysphagia, and we recommend its use in all patients after intubation.
